The article "Revealing the Moderating Role of Organizational Support in HR Professionals’ Competencies, Willingness, and Effectiveness Relationship: Empirical Evidence From a Developing Economy" was published in 2022. Journal: Front Psychol.

# Revealing the Moderating Role of Organizational Support in HR Professionals’ Competencies, Willingness, and Effectiveness Relationship: Empirical Evidence From a Developing Economy

**DOI:** 10.3389/fpsyg.2022.756255

**Published:** 2022-07-05

**Authors:** Aqeel Ahmad, Muhammad Fareed, Mohd Faizal Mohd Isa, Sri Sarah Maznah Mohd Salleh

**Affiliations:** ^1^Faculty of Management Studies, University of Central Punjab (UCP), Lahore, Pakistan; ^2^School of Business Management, Universiti Utara Malaysia, Sintok, Malaysia; ^3^Faculty of Applied and Human Sciences, Universiti Malaysia Perlis, Kangar, Malaysia; ^4^Centre of Excellence for Social Innovation and Sustainability, Universiti Malaysia Perlis, Sintok, Malaysia

**Keywords:** HR professionals’ effectiveness, HR professionals’ competencies, HR professionals’ willingness, organizational support, banking sector

## Abstract

Human resources management is essential to ensure the success of any organization which is based on the belief that an organization gains competitive advantage by using its people effectively and efficiently. But HR professionals need organizational support to make the employees more committed and passionate about their work. In this study, the researchers aim to examine the moderating effect of organizational support in the relationship between human resource (HR) professionals’ competencies, HR professionals’ willingness, and HR professionals’ effectiveness. HR Professionals’ competencies such as credible activist, talent manager, culture and change steward, strategy architect, business ally, and operational executor nurture HR professionals’ effectiveness. Besides, HR professionals’ willingness is a significant predictor of HR professionals’ effectiveness. To test the relationships, the researcher collected data through survey questionnaire from 183 managers from commercial banks of Pakistan. For statistical analysis, Partial least squares-structural equation modeling (PLS-SEM) is used to analyze the data and test the hypotheses. The findings reveal the positive and significant impact of HR professionals’ competencies and HR professionals’ willingness on HR professionals’ effectiveness. Additionally, the moderating impact of organizational support was also significant among HR professionals’ competencies, HR professionals’ willingness, and HR professionals’ effectiveness relationship. The study contributes in the literature of HR professionals’ effectiveness and organizational support in the banking sector of local context. The study also discusses the implications and future directions. One of them is that the research framework provides guidelines for HR professionals about what competencies are needed to enhance HR professional effectiveness. The present study recommends HR professionals of the banking sector to be involved in strategic planning and implementation in their organization.

The article "Revealing the Moderating Role of Organizational Support in HR Professionals’ Competencies, Willingness, and Effectiveness Relationship: Empirical Evidence From a Developing Economy" was published in 2022. Journal: Front Psychol.

## Introduction

In today’s technological era, the paradigm of agricultural, industrial, and service economy has shifted to a knowledge-based economy, which has also transformed the roles and functions of the human resource (HR) in organizations (García-Carbonell et al., 2018; Nam and Lee, 2018; Szierbowski-Seibel and Kabst, 2018). HR functions were conventionally handled by general administration, and day-to-day HR operations were considered as the primary role (Novicevic and Harvey, 2001; Kazlauskaite and Bučiuniene, 2010). Over the decades, HR has taken on multiple managerial roles, including strategic focus, people-orientation, and operational efficiency (Truss, 2009; Kim and Ryu, 2011; Lo et al., 2015).

This shift in HR practice has led to a distinct identity of HR employees as HR professionals. Ulrich et al. (2009) have reiterated that business challenges have become more complex, creating a demand for a higher level of competent, skilled, and responsive workforce in the organizations. Al-Busaidi et al. (2021) believe that any organization’s most important asset has its employees. They are the key contributors to the performance of the organization. These employees tend to have exceptional HR attributes like core HR competencies that contribute to an organization’s success (Lawler and Mohrman, 2003). These are a set of characteristics contributing to HR professionals’ effectiveness that enable an organization to carry out its business strategies in a competitive market (Long, 2008; Mariappanadar, 2019). A competency model involving knowledge, skills, capabilities, and behaviors enables HR professionals to perform a job or sustain the desired organizational culture and growth (Ulrich et al., 2009).

This study uses Resource-Based View (RBV) theory of J. Barney as underpinning theory. The theory focuses on internal strengths and weaknesses of an organization and argue that a resource fulfilling VRIN (valuable, rare, imperfectly imitable, and non-substitutable) condition will be effective resource to gain competitive advantage in the market (CIHAN-OKSUZOGLU & GUROL). Based on this argument, the theoretical background of the study has been formed. This study states that HR competencies and willingness being significant resource cause significant impact on effectiveness of HR professionals.

HR professional competencies enhance HR professional effectiveness (Becker et al., 1997; Huselid et al., 1997a). Most empirical research on HR professionals’ competencies has been developed and tested in countries like Malaysia, the United States, Taiwan, and European Countries (Boselie and Paauwe, 2005; Han et al., 2006; Ulrich et al., 2007; Sang, 2009). These previous studies on HR professional competencies have been carried out mostly in the manufacturing firms (Han et al., 2006; Ulrich et al., 2007; Sang, 2009; Abdul Hamid et al., 2011) with research on the financial sector covering is very limited. Banking sector is an important financial sector for the economic life of developed and less developed countries. It has witnessed a remarkable progress recently (Mohd Ali and Sovaniski, 2021). As far as banking sector of Pakistan is concerned, it is facing a lot of challenges and it is research deficient sector (Ali et al., 2021). Over the past decade, the reforms initiated by State Bank of Pakistan (SBP) have identified the lack of competencies of HR Professionals as an impediment in the face of the growth potential of the banking sector (Ahmad et al., 2015). Studies of Budhwar and Debrah (2013) and Siddiquee (2003), cited in Ahmad et al. (2019), investigated the HR practices in south Asian countries and directed that HR performance in these countries is below the strategic level and require other professional practices. Particularly, Pakistan has been identified as research deficient in the HRM discipline (Aycan et al., 2000). The banking sector of Pakistan needs HR implementation due to high competition globally (Qureshi et al., 2010). But the banking sector of Pakistan faces many challenges in implementing HR practices, especially in recruitment and selection and training and development. The Non-performing loan (NPL) has been a growing concern for bank managers and credit officers, which negatively impacts the banking sector of Pakistan (Jameel, 2014). State Bank of Pakistan (2019) revealed an increase in NPL from Rs. 623.6 billion in 2018 to 768 billion in 2019. NPL show lack of competency of HR manager who was not able to hire a competent employee that can help reducing NPL. Many experts believed that the increase of bank’s NPL is due to the lack of trained staff in debt disbursement and collection and incompetency of HR professionals in their role of recruiting appropriate talent (Ahmad et al., 2013; Gupta and Jain, 2014; Fareed et al., 2016). Therefore, the HR professional’s competencies and their professional effectiveness are highly under scrutiny in the banking sector of Pakistan, and there is a dire need to empirically test the factors contributing to HR professional effectiveness in this context (Awan and Farhan, 2016; Fareed et al., 2016). These include HR competencies and willingness.

The article "Revealing the Moderating Role of Organizational Support in HR Professionals’ Competencies, Willingness, and Effectiveness Relationship: Empirical Evidence From a Developing Economy" was published in 2022. Journal: Front Psychol.

In addition, El-Kassar et al. (2022) pointed out that positive employee behavior and commitment were somehow linked with organizational support. If the employees perceived that the organization acknowledged their accomplishments, they might be passionate. Mathis and Jackson (2010) highlighted organizational support as a critical factor in effectively aligning HR professionals’ competencies with the needs of an organization. Sharif and Ahmad (2009) also proposed in their study that organizational support has some moderating impact among behavioral variables in an organization. Hence, the purpose of this study is to examine the moderating relationship of organizational support between human resource (HR) professionals’ competencies, HR professionals’ willingness, and HR professionals’ effectiveness. Multiple studies use organizational support as mediating variable to explore its impact on performance (Desa and Asaari, 2020; Côté et al., 2021). The moderated effects of organizational support are still to be explored. This study fulfills this gap.

## Literature Review and Hypotheses Development

### HR Professionals’ Competencies and HR Professionals’ Effectiveness

Ulrich et al. (2010) define competencies as the knowledge, skills, and behaviors demonstrated by individuals in getting their tasks done. HR competencies help to enhance employee satisfaction (Daguplo et al., 2019). A study by Martina et al. (2012) also defined it as the act of asserting one’s real working potential. These are a combination of employee’s attributes like knowledge, skills, and abilities. These further contain personality features that enable HR professionals to be useful members of the organization (Daguplo et al., 2019).

Similarly, many authors proved that competencies are relative to employees’ characteristics (knowledge, skills, behavior, attitude, aptitudes, and social motives) which are linked to effective and advanced job performance (Dubois and Rothwell, 2004; Ellis, 2014; Fareed et al., 2019, 2020). HR effectiveness can be defined as the outcome of HR activities. The HR activities include HR competency, manager support, and compensation planning and strategy contributions.

Moreover, competencies refer to the ability to perform a particular activity, have certain general and specific knowledge, abilities, skills, and attitude to be qualified in a specific work-related area. Therefore, we can argue that competencies are required to achieve the required level of effectiveness. According to Heinsman et al. (2007), HR competencies have become the leading construct in HRM research to improve an employee’s performance. Aitchison (2007) also pointed out that the main obstacle for HR professionals to perform effectively in organizations is their lack of competencies.

The article "Revealing the Moderating Role of Organizational Support in HR Professionals’ Competencies, Willingness, and Effectiveness Relationship: Empirical Evidence From a Developing Economy" was published in 2022. Journal: Front Psychol.

A significant modification of HR professional competencies by Ulrich et al. (2007) and colleagues suggested six competencies domains: credible activist, cultural and change steward, talent manager/organizational designer, strategic architect, business ally, and operational executor. Some of these competencies, including culture and change steward (CCS), talent manager/organization designer (TMOD), and strategic architect (SA), enable HR professionals’ to develop organizational capabilities, which in turn can create competitive advantage (Ulrich and Grochowski, 2012). However, Business ally (BA) and operational executor (OE) do not differentiate an organization or an employee, but knowledge and competency in these areas are required for better performance. This version of the Ulrich et al. (2007) model is deemed the most relevant to the current business environment and directly related to HR professionals in the 21st century. Based on this argument, this study examines HR professional competencies and their influence on professional’s effectiveness by using Ulrich model and the level of effectiveness where organizational support can moderate this relationship.

### Credible Activist and HR Professionals’ Effectiveness

According to Grossman (2007), credible activist (CA) competency is the top indicator of HR professional performance. This competency is at the heart of what it takes to be an effective HR professional. Ulrich et al. (2010) argued that the HR professional needs to be both credible (respected, admired, and listened to) and active (offers a point of view and takes challenging assumptions). Some have called this “HR with an attitude.” HR professionals who are credible but not activists are admired but have little impact. Activists who are not credible have the idea that no one implements. The credible means that HR professionals must be respected, admired, listened, and honored and activist means that he should be active to offer his point of view and meet challenges. Those who are Activist but not credible may not be listened to even though they have good ideas. The competency, Credible Activist, dominates all other competencies as it serves as the heart of competencies (Enkhjav et al., 2020). Ulrich et al. (2009) stated that “Credibility” moves the HR professional up the people axis, and activism moves them up the business axis. Both are involved in HR professional performance.

Since HR professionals work with the human side of the business, they need to have strong interpersonal skills. Credible Activists create an environment of trust that leads to results in optimistic working relationships with all employees of the organization. Ulrich et al. (2009) found that Credible Activists created a strong relationship between employee effectiveness and business performance. Selmer and Chiu (2004) identified that HR professionals with credible activist competency could become more useful for their organizations’ business success. Inyang (2010) argued that HR professionals should act with integrity in all business dealings and honor a personal commitment. They need to develop inter-relationships with all the employees of the organization. Highly effective HR professionals are focused both equally on the organization’s business and HR-related needs. In general, the credible activist domain has the most significant influence on HR professionals’ effectiveness. Hence, we can hypothesize that as:

*H1*: Credible activist has a significant positive impact on HR professionals’ effectiveness.

The article "Revealing the Moderating Role of Organizational Support in HR Professionals’ Competencies, Willingness, and Effectiveness Relationship: Empirical Evidence From a Developing Economy" was published in 2022. Journal: Front Psychol.

### Talent Manager/Organization Designer and HR Professionals’ Effectiveness

Attracting, developing, and retaining talent are the second most eminent functions of HR professionals’. According to Ulrich et al. (2009), the most effective HR professionals’ are both talent managers and organization designers. Talent management focuses on competency requirements and how individuals enter and move up, across, or out of the organization. An organization designer focuses more on how an organization incorporates capability into the structure, processes, and policies that shape the working of an organization. Grossman (2007) argued that the appreciation or depreciation of the value of a human asset depends on the intelligence and effectiveness of an organization’s design. Similarly, Kaplan and Norton (2004) also found that it is difficult to reach a high sustainable performance without the alignment of an organizational design and talent placement. It does not matter how talented the employees are if the underlying processes and structures are misaligned. Therefore, it is a vital area for HR professionals’ to be competent where they have to take the lead to engage their employees and enable them to contribute to the organizational performance (Morgan and Jardin, 2010). According to Dhanpat et al (2020), talent manager is responsible for knowing what skills are required to the employees and how to improve those skills. Talent Management means the knowledge of customer requirement, strategy, and integration of each other. The organizational Designer means the ability of HR professional to design the policies and structure of the organization or shaping the organization how it works. Talent Management and Organizational designing work together and success cannot be sought in long run by the organization without their active integration (Payne, 2010; Theys and Schultz, 2020).

The article "Revealing the Moderating Role of Organizational Support in HR Professionals’ Competencies, Willingness, and Effectiveness Relationship: Empirical Evidence From a Developing Economy" was published in 2022. Journal: Front Psychol.

Developing talent ultimately leads to higher retention and productive employees. Organizational structure refers to the structure of an organization to achieve its desired goals. HR professional is not only about the talent or an organization design; it is about both of them interacting simultaneously. Ulrich et al. (2008) argued that talent with no supporting organization design might not be sustained, and an effective organization design may not deliver results without talented employees. HR professionals ensure that a company’s talent management and organizational capabilities are aligned with customer requirements and strategy by integrated with each other and worked effectively and efficiently. Building HR professional competencies in the Talent Manager/Organization Designer domain is a significant way to make the HR professionals’ to be effective. HR professionals need to balance between getting and developing the right talent and ensuring that the organization’s structure is conducive to delivering the desired organization capabilities. Kaliannan et al. (2016) suggested that an HR professional as a talent manager is responsible for recruiting, managing, analyzing, promoting, and retaining the employees in their organization.

Ellehuus (2012) found that HR professionals’ have talent management competency, which helps them generate more profit and enhance their employees’ performance by up to 25 percent. Many managers understand the importance of this competency, and most of them fail to link strong talent management/organization designer competency and the success of their business. HR professionals can effectively perform as a talent manager/organization designer competency for their organization’s growth. This study thus hypothesized that as:

*H2*: Talent manager/organization designer has a significant positive impact on HR professionals’ effectiveness.

### Culture and Change Steward and HR Professionals’ Effectiveness

Culture and change became a common buzzword in the late 20th century. The 1980s and 1990s brought a dramatic era of downsizing, mergers, acquisitions, and restructuring for many organizations. Culture and change have been acknowledged as an influential factor in examining the performance of an organization (Wilkins and Ouchi, 1983; Jones et al., 2005). According to Dhanpat et al (2020) and Junita (2021), the change agent is one who embraces change in the organization, responds actively to the change, and lets people know how to deal with the change. Ulrich et al. (2008) argue that culture has been an essential feature in HR competency studies since 1997. Restructuring of the HR system is often implemented when organizations undergo structural and cultural changes. Wright and Snell (1998) suggested that when companies respond to dynamic environments, the HR professionals are expected to drive their efforts to build flexible organizations. HR professionals first develop practices in a way that can be accepted; second, expand the skill sets of their employees; and finally, develop their employees’ behavioral flexibility. It is challenging to become a competent culture and change steward. When HR professionals lead an organizational change, the chances are high that they will send out confusing rather than coherent and consistent messages to the employees. Culture is a not a single event but a series of activities. Meeting external customer expectations with internal employee and organization behaviors is termed as culture. Culture steward is HR professionals who respect the old culture and help to shape the new culture. They direct managers to reflect the culture by their actions. In reality, they make the culture. Successful HR professionals help make culture happen and develop discipline to make changes happen in the organization (Sabuhari et al., 2020; Febriyarso and Ruslan, 2021).

The article "Revealing the Moderating Role of Organizational Support in HR Professionals’ Competencies, Willingness, and Effectiveness Relationship: Empirical Evidence From a Developing Economy" was published in 2022. Journal: Front Psychol.

Ulrich et al. (2008) found that effective HR professionals clearly understand the culture required to deliver the business strategy and communicate the desired culture broadly and frame it to engage employees. Effective HR professionals develop their organizations’ potential for change and transform that potential into effective change processes and structure. Edgley-Pyshorn and Huisman (2011) emphasized that HR professionals have to take the role of teacher, guiding and facilitating their employees to perform better in the cultural change process. They can motivate all employees of their organization and adjust their behavior to fit-in the new culture. HR professionals must work with the management team and other key individuals to ensure the sustainability of the cultural change. Any organization embark on a culture change program should enlist HR professionals in defining and enacting the culture. When HR professionals have the skills to make culture real, they help their organization to become competitive and this competency therefore becomes more significant and effective for HR professionals in many organizations (Wiley, 2010; Ahmad et al., 2012). Thus, it can be hypothesized that as:

*H3*: Culture and change steward has a significant positive impact on HR professionals’ effectiveness.

### Strategy Architect and HR Professionals’ Effectiveness

The strategy architect is one who has ability to clarify the external trends and use them according to the internal actions and finally communicates its effect on human capital (Dhanpat et al., 2020). Strategic focus across all functional areas is the key to success. HR professionals are expected to safeguard organizational policies and strategies. While exploring the psychological frames of HR professionals, Labedz and Lee (2011) found that these professionals do not have a strategic outlook yet have shown people-oriented behaviors. Ulrich et al. (2008) argue that HR professionals must thoroughly master the business’s strategic architecture in which they work. They need an in-depth appreciation of the business portfolio, making each business distinctive in the customers’ eyes. HR professionals must understand the business strategy and align HR practices with it. It includes identifying the problems central to the business strategy, recognizing marketplace trends and their impact on the business, and translating the strategic direction into annual business and HR initiatives. According to Brockbank et al. (2012), the HR professionals must also be aware of the global business context, and they should apply this knowledge in developing a personal vision for the future of the organization. They need to develop customer-focused business strategies and translate the business strategy into annual business plans and goals. The strategy Architect competency helps to contribute overall business strategies. A Strategy Architect knows the art of changing negative to positive and how to formulate strategy or use strategic tools to keep progress. Leaders and HR professionals contribute significantly to strategy by integrating internal stakeholder and external stakeholder expectations (Junita, 2021).

The article "Revealing the Moderating Role of Organizational Support in HR Professionals’ Competencies, Willingness, and Effectiveness Relationship: Empirical Evidence From a Developing Economy" was published in 2022. Journal: Front Psychol.

Moreover, HR professionals have to take responsibility for the process of developing strategy regularly. However, they cannot contribute at the strategic level in their organizations because it is perceived that they lack the competency to work at the strategic level (Edgley-Pyshorn and Huisman, 2011; Reilly, 2012). Therefore, HR professionals need to focus on a vision on how the organization can “win” in the marketplace, now and in the future. They can then play an active part in establishing an overall strategy to deliver on this vision. It would require them to recognize business trends and how these will impact the business, thus forecasting potential obstacles to success and facilitating strategic clarity. This linkage helps make customer-driven business strategies real to the employees of the company (Ulrich et al., 2007). Similarly, Inyang (2010) argued that HR professionals must think about how they can contribute as strategic resources and contribute to organizational growth. Therefore, we can hypothesize that as:

*H4*: Strategy architect has a significant positive impact on HR Professionals’ effectiveness.

### Business Ally and HR Professionals’ Effectiveness

This competency states that HR Professionals must have knowledge of his business, his customers, and products to successfully achieve the objectives of business. They must have understanding of all departments of business i.e., Marketing, Sales, Accounts, and research to help the business to earn money (Sharma and Sakpal, 2019). According to Ulrich et al. (2009), the competency of Business Ally has shifted dramatically from the last few decades. At first, “understanding the business” was very significant for an HR professional to be perceived as competent. But, in 2002, it was found by Ulrich et al. (2007) for the first time that “understanding the business” is one of the weakest statistical predictors of an HR professional overall competence. Businesses succeed by setting goals and objectives that respond to external opportunities and threats. HR professionals contribute to a business’s success by knowing the social context or setting in which their business operates. They also know how the business makes money, in terms of who the customers are, why they buy the company’s products or services.

Payne (2010) conducted their study in the Midwest region of the United States and found that HR professionals must develop competencies, particularly those that are business-related. Business-related competency is the need of the day. Ulrich et al. (2008) stated that HR professionals are increasingly expected to contribute directly to the success of their organizations’ business, and businesses succeed by profitable responding to changing external conditions. Therefore, HR professionals help drive the business’s success by knowing the broader setting in which the business operates. In addition, HR professionals must understand the value chain of the business, how it makes money, how it coverts less-valuable inputs into more-valuable outputs, and how resources within the company are arranged to deliver on customer expectations.

Furthermore, when HR professionals speak intelligently about a balance sheet or make recommendations based on market conditions, their credibility increases. This credibility allows them opportunities to participate in increasingly more strategic discussions at all levels of the organization. Being a business ally is not about memorizing only the financials of an organization but rather about being aware of what is going on around them. Inyang (2010) argued that HR professionals must understand the organization’s business direction and its competitive position in the market. HR professionals must have business-related competency, which can become more effective. Accordingly, it can be hypothesized that as:

*H5*: Business Ally has a significant positive impact on HR professionals’ effectiveness.

The article "Revealing the Moderating Role of Organizational Support in HR Professionals’ Competencies, Willingness, and Effectiveness Relationship: Empirical Evidence From a Developing Economy" was published in 2022. Journal: Front Psychol.

### Operational Executor and HR Professionals’ Effectiveness

This competency states that HR professional has to hold the operations of any organization so he/she needs to be able to draft, adapt, and implement policies. If there is flaw in the policies of HR professional, it spoils his credibility. These skills are ranged in HR activities as Transactional or legacy. The operational activities like policies which need to be drafted, adapted, and implemented and hiring and training of employees are all vital so they are highly needed to an HR professional (Khabibullina, 2019).

Some scholars have emphasized the importance of organization operational execution as a competitive edge in service organizations, especially in banks (Wilkinson et al., 2009). Roth and Van Der Velde (1991), for example, suggested a service strategy must address how operations will support and network with the competitive weapon of a business. In the past day-to-day activities and policy, issues were the prime responsibility of the personnel department (Anthony et al., 1999). The personnel department managed the paperwork, employee hiring, firing, paying, and promoting. Operational implementations of HR activities are administrative in nature. The personnel department focused on the terms and conditions of work and the running of the administrative systems to assist the employees in performing their duties properly (Ulrich et al., 2008).

HR professional as an operational executor is responsible for HR procedures that need to be documented and implemented. Employees also have many administrative needs (e.g., to be paid, relocated, hired, and trained). It revolves around the HR professional’s ability to execute the operational aspects of managing people and organizations. HR professionals ensure that these basic needs are efficiently dealt with through technology and shared services. Furthermore, HR professionals must develop working relationships with line managers and employees and consider their suggestions for better operational execution. The HR professional is accountable for ensuring these fundamental needs are effectively met (Ulrich et al., 2009). Hence, the following can be hypothesized.

*H6*: Operational executor has a significant positive impact on HR Professionals’ effectiveness.

### HR Professionals’ Willingness and HR Professionals’ Effectiveness

The word “Will” is associated with intrinsic motivation to be useful or not. Willingness is made up of the belief, attitudes, and intentions of the employees involved in knowledge-related activities (Smith and McLaughlin, 2004). Smith and McLaughlin (2004) further argued that if the will is combined with employees’ competencies and capabilities, then personal performance will go up. If HR professionals lack the willingness and motivation to contribute their knowledge and expertise, they may not be effective (Raza et al., 2020). One way by which HR department can add value to its organization is that HR professionals be willing to actively contribute to HRM strategies and their implementation.

The article "Revealing the Moderating Role of Organizational Support in HR Professionals’ Competencies, Willingness, and Effectiveness Relationship: Empirical Evidence From a Developing Economy" was published in 2022. Journal: Front Psychol.

Kurz and Bartram (2002) argued that activities and roles could be performed more innovatively if managers are willing. Currie and Kerrin (2003) claimed that employees lack the willingness and motivation to contribute their knowledge if competent managers are not appraised justly, resulting in project failures. Another study by Chen and Silverthorne (2005) also reported that competency and willingness affect each other (positively or negatively) while employees’ willingness will enhance the assigned task’s efficiency and effectiveness because of increased competency. Analoui (1999) also argued that competencies alone could not be adequate for managerial effectiveness. There is also a need for employee willingness, which will play a vital role in their effectiveness. Further, Raza et al. (2020) suggested to study employees’ willingness to perform with employee effectiveness as they have highlighted employee willingness is a new concept and it should be studied in future studies. It leads to the following hypothesis:

*H7*: HR professionals’ willingness has a significant positive impact on HR professionals’ effectiveness.

### The Moderating Role of Organizational Support

Organizational support refers to the beliefs of an employee that the organization values his contribution toward the success of organization and also cares about his welfare. This is actually a support from organization to the employee which shows the significance of the employee in the eye of organization. The behavior of an employee is affected by this perception. This is an exchange relationship between employee and organization (Desa and Asaari, 2020). Organizational support for employees in various ways has been initiating interest in management scholars (AL-Abrrow, 2018). It is now well accepted among various scholars and as one vital factor playing a significant role in improving the employees’ and organizations’ effectiveness (Shore and Wayne, 1993; Yoon and Lim, 1999). It is the feeling that organization cares for the employee (Alnaimi and Rjoub, 2019). HR professionals may not be effective in performing their role if they lack adequate staff, the latest technology, financial resources, and top management empowerment. Organizational support tends to reduce adverse job outcomes and reduce turnover intentions (Baranchenko et al., 2020). It reduces negative employee outcomes such as knowledge hiding behavior and extra role behavior as it initiates a sense of social exchange (Alnaimi and Rjoub, 2019).

The article "Revealing the Moderating Role of Organizational Support in HR Professionals’ Competencies, Willingness, and Effectiveness Relationship: Empirical Evidence From a Developing Economy" was published in 2022. Journal: Front Psychol.

In many studies on relationships in the management literature, the intervening variable or moderating variable has been found to play some role (Chenhall and Brownell, 1988; MacKinnon et al., 2002; Stephen, 2017). Sharif and Ahmad (2009) found that organizational support has a moderating role in studying behavioral variables in organizations. The importance of organizational support as an intervening variable in behavioral studies is further enhanced by earlier researchers (Schermerhorn, 1975). Employees’ performance is mainly a result of organizational support because it enables them to utilize their competencies effectively. Baranchenko et al. (2020) considered and realized the moderating impact of organizational support between employability and turnover intentions. AL-Abrrow (2018) also identified that organizational support serves the moderator’s role between organizational politics and silence. Thus, this study is also interested in investigating the moderating effect of organizational support on HR professionals’ effectiveness.

Furthermore, the HR sub-functions are related to recruitment and selection, training and development, and performance-based reward system. If these are supported relatively and adequately, they will affect competency building and professionals’ willingness such that their effectiveness will be enhanced accordingly. According to Mathis and Jackson (2010), many factors affect the performance of individual employees, including their abilities, efforts expended, and the organizational support they receive. Kane et al. (1999) found that HRM effectiveness can be attained by organizational support. At the same time, Black et al. (2003) argued that it is challenging for HR professionals to get adequate support from their organization due to the lack of financial investment in this particular area. Organizational support not only satisfies employees’ motivation to take their job seriously but may also affect the employees’ willingness (Lin and Lin, 2011). According to Desa and Asaari (2020), the employees who think that their organization support them, they perform better than those who feel they are not supported by the organization. Well-coordinated management practices can also enhance the effectiveness of the employees particularly, and as such organizational support is highly effective in firms that are service-oriented like banks. It leads to research the following hypothesis (Figure 1):

**Figure 1:** Research model.

The article "Revealing the Moderating Role of Organizational Support in HR Professionals’ Competencies, Willingness, and Effectiveness Relationship: Empirical Evidence From a Developing Economy" was published in 2022. Journal: Front Psychol.

*H8*: Organizational Support moderates the relationship between HR professionals’ competencies, HR professionals’ willingness, and HR professionals’ effectiveness.

Theoretically, all the study hypotheses are supported by the resource-based theory of barney. Barney discusses that organizations should identify and develop unique assets to get maximum results. As we discussed, employees are the critical assets of any organization. To get a competitive advantage, organizations need competent employees who are not replaceable and have all the qualities of VRIN. All the HR Professional’s competencies and HR professionals will have a significant and positive impact on HR Professional’s Effectiveness. Organizational support moderates the relationship between HR professionals’ competencies, HR professionals’ willingness, and HR professionals’ effectiveness.

## Research Methodology

The survey questionnaires were collected from the managers of the private sector banks of Pakistan. The total number of branches of all banks operating in Pakistan stood at 14,197, out of which 10,835 (represented about 75.32%) branches belonged to the private sector banks (State Bank of Pakistan, 2019). Before distributing the final questionnaires, it was reviewed by two professionals and three academicians to determine the appropriateness of the instrument within the Pakistani context, especially in the banking sector environment. Based on their suggestions, several items from the instrument were excluded as they are more suitable for studies in developed countries. Besides, a pilot study involving 35 branch managers from five different private banks of Pakistan was conducted. The respondents reported that the questionnaire is easy to complete. The results of the pilot study sustained that no changes are necessary for the questionnaire. Thus the questionnaire is considered reliable and internally valid.

To collect the current study’s actual data, 370 survey questionnaires were distributed through the snowball sampling technique. Every set of questionnaires was attached with a cover letter stating the objective of the study, instructions, confidentiality of the information or data, and anonymity of the respondents. In the snowball sampling approach, the researchers distributed questionnaires to the individual manager with whom the researchers had initial contacts and formed the first tier of Snowballing references. From 370 questionnaires, 187 were returned, resulting in a response rate of 50.5%. Out of the 187 returned questionnaires, four questionnaires were incomplete and excluded from analysis; hence, 183 questionnaires were analyzed. From 183 responses, 77% were male, and 23% were female. In terms of their managerial position, 38.8% of respondents worked as a branch manager, 33.9% were as an operational manager, 9.8% were a customer relationship manager, 10.9% were as a credit manager, and 6.6% were as a regional manager. Moreover, concerning their level of education, 3.3% had MS/MPhil degree, 80.3% had a Master’s degree, and 16.4% had a bachelor’s degree.

The article "Revealing the Moderating Role of Organizational Support in HR Professionals’ Competencies, Willingness, and Effectiveness Relationship: Empirical Evidence From a Developing Economy" was published in 2022. Journal: Front Psychol.

### Instrumentation

The constructs for the present study were adapted from the model of Ulrich et al. (2007). In HR professionals’ competencies, 9 items were used for measuring Credible Activist, 10 items for Talent Manager / Organization Designer, 8 items for Culture and Change Steward, 12 items for Strategy Architect, 11 items for Business Ally, and 8 items for Operational Executor. Sample items for HR professionals’ competencies are credible activist “HR professionals in our bank respond promptly to our issues,” talent manager “HR professionals in our bank are able to promote talented employees,” culture & change steward “HR professionals in our bank take a proactive role in bringing about change,” strategy architect “HR professionals in our bank translate business strategy into annual business initiatives,” business ally “HR professionals in our banks are aware of the social issues having an impact on the banks business,” and operational executor “HR professionals in our bank are good at managing the labor policies and procedures.” Han et al. (2006) and Sharif and Ahmad (2009) scales were adapted to measure HR’s professional willingness (7 items), Organizational support (10 items), and HR’s professional effectiveness (11 items). Sample items are, HR professionals’ willingness “HR professionals in our bank are self-motivated to take proactive actions” organizational support “HR department has been provided with adequate training budget in order to enhance the competency level of their HR professionals” and HR professionals’ effectiveness “HR professionals in our bank have given value-added contributions to our bank’s operational performance.” All the instrument items were measured through 5 points Likert Scale ranging from 1 (Strongly disagree) to 5 (Strongly agree) by using the English language.

## Data Analysis and Results

### Common Method Variance and Normality of the Data

*Post-hoc* Harman single factor test was applied to check common method variance (Podsakoff et al., 2003). The principal component analysis was run at which all measurement items were included for factor analysis and examined the un-rotated solution. A single factor of an un-rotated solution of principal component analysis explained 32.92% of the variance, which was lower than 50%. Hence, it indicates the absence of common method variance in our study. The skewness values of all instrument items in our study ranged from −0.022 to −1.148 and kurtosis values from 0.090 to 2.116, which proved that the data had followed the conditions of normality (Kline, 2015).

The article "Revealing the Moderating Role of Organizational Support in HR Professionals’ Competencies, Willingness, and Effectiveness Relationship: Empirical Evidence From a Developing Economy" was published in 2022. Journal: Front Psychol.

### Measurement Model

The partial least squares-structural equation modeling technique (PLS-SEM) was applied in a statistical software Smart PLS to test the measurement and structural models. The researcher uses the PLS-SEM because it handles very complex models with many indicators and constructs, estimate normatively specified constructs, able to deal with small sample sizes, and determinate latent variable scores, which can be applied in subsequent analyses. Before testing the structural model, a measurement model was assessed by computing convergent and discriminant validity. Outer loadings of construct items found with less than 0.40 were deleted from the model. This research has established the threshold criteria for outer loadings given by Hair et al. (2016). According to this criteria items’ loadings which have been retained for testing the model ranged between 0.416 and 0.919 which is considerably accepted in exploratory research because retaining these items have competed the threshold criteria of AVE (0.5) and CR (0.7) proposed by Fornell and Larcker (1981), Bagozzi and Yi (1988), and Hair et al. (2016). Generally, indicators with loadings between 0.40 and 0.70 should only be considered for removal from the scale if deleting this indicator leads to an increase in composite reliability above the suggested threshold value. Another consideration in the decision to delete indicators is the extent to which their removal affects validity. Weaker indicators are sometimes retained on the basis of their contribution to content validity (Hair et al., 2011). Only if an indicator’s reliability is low and eliminating this indicator goes along with a substantial increase of composite reliability, it makes sense to discard this indicator (Henseler et al., 2009). Table 1 shows the findings of CFA where Cronbach’s Alpha and Composite Reliability values of all variables are greater than 0.7. Moreover, loadings of all instrument items and Average variance extracted (AVE) values are also higher than the recommended threshold of 0.50 which confirm the convergent validity as evident by Figure 2 (Hair et al., 2016).

The article "Revealing the Moderating Role of Organizational Support in HR Professionals’ Competencies, Willingness, and Effectiveness Relationship: Empirical Evidence From a Developing Economy" was published in 2022. Journal: Front Psychol.

**Table 1:** Results of convergent validity and reliability.

Constructs	Measurement items	Item loadings	Cronbach’s alpha	Composite reliability	AVE
Business Ally	BA2	0.580	0.779	0.839	0.50
	BA3	0.769			
	BA4	0.919			
	BA9	0.720			
	BA10	0.547			
	BA11	0.510			
Credible Activist	CA1	0.669	0.840	0.878	0.549
	CA2	0.856			
	CA3	0.815			
	CA7	0.720			
	CA8	0.672			
	CA9	0.691			
Culture & Change Steward	CCS1	0.784	0.896	0.917	0.580
	CCS2	0.688			
	CCS3	0.693			
	CCS4	0.751			
	CCS5	0.854			
	CCS6	0.747			
	CCS7	0.805			
	CCS8	0.755			
HR Professionals’ Effectiveness	HRPE1	0.872	0.867	0.905	0.623
	HRPE2	0.842			
	HRPE3	0.875			
	HRPE7	0.801			
	HRPE10	0.830			
	HRPE11	0.416			
HR Professionals’ Willingness	HRPW1	0.831	0.910	0.929	0.653
	HRPW2	0.805			
	HRPW3	0.756			
	HRPW4	0.855			
	HRPW5	0.846			
	HRPW6	0.901			
	HRPW7	0.635			
Operational Executor	OE1	0.678	0.872	0.896	0.530
	OE2	0.850			
	OE3	0.805			
	OE4	0.775			
	OE5	0.839			
	OE6	0.416			
	OE7	0.793			
	OE8	0.549			
Organizational Support	OS1	0.606	0.893	0.913	0.513
	OS2	0.639			
	OS3	0.736			
	OS4	0.779			
	OS5	0.747			
	OS6	0.664			
	OS7	0.715			
	OS8	0.700			
	OS9	0.802			
	OS10	0.752			
Strategy Architect	SA1	0.642	0.892	0.914	0.539
	SA2	0.697			
	SA3	0.809			
	SA6	0.802			
	SA8	0.753			
	SA9	0.800			
	SA10	0.749			
	SA11	0.607			
	SA12	0.720			
Talent Manager/Organization designer	TMOD1	0.752	0.877	0.899	0.502
	TMOD3	0.693			
	TMOD4	0.890			
	TMOD5	0.611			
	TMOD6	0.722			
	TMOD7	0.706			
	TMOD8	0.618			
	TMOD9	0.803			
	TMOD10	0.509			

**Figure 2:** Measurement model.

Fornell-Larcker criterion and cross-loading were applied to measure discriminant validity (Fornell and Larcker, 1981; Hair et al., 2017). Table 2 shows the results of discriminant validity, where the square roots of AVE of all variables are greater than their correlation.

**Table 2:** Discriminant validity.

	BA	CA	CCS	HRPE	HRPW	OE	OS	SA	TM/OD
BA	**0.707**								
CA	0.698	**0.741**							
CCS	0.673	0.681	**0.762**						
HRPE	0.694	0.713	0.732	**0.789**					
HRPW	0.701	0.724	0.681	0.787	**0.808**				
OE	0.586	0.636	0.613	0.587	0.696	**0.728**			
OS	0.699	0.671	0.610	0.709	0.706	0.567	**0.716**		
SA	0.513	0.707	0.719	0.693	0.723	0.560	0.664	**0.734**	
TM/OD	0.698	0.601	0.681	0.622	0.695	0.650	0.630	0.678	**0.709**

### Structural Model

For testing hypotheses in the relationship model, beta values (*β*), t statistics, and values of *p* were examined in SmartPLS software. Figure 3 and Table 3 reveal that Business Ally (*β* = 0.093^*^, *t* = 2.007), Credible activist (*β* = 0.143^***^, *t* = 3.159), Operational Executor (*β* = 0.177^***^, *t* = 4.03), Strategy Architect (*β* = 0.163^**^, *t* = 2.332), Talent Manager/Organization Designer (*β* = 0.142^**^, *t* = 2.267), Organizational Support (*β* = 0.078^**^, *t* = 2.331), and HR Professionals’ Willingness (*β* = 0.667^***^, *t* = 20.132) were positively and significantly associated with HR’s professional effectiveness. Whereas, Culture and Change Steward also had a positive but statistically insignificant relationship with HR’s professional effectiveness (*β* = 0.10, *t* = 1.434). The study found the most significant relationship of HR professional’s effectiveness was with HR Professionals’ Willingness.

The article "Revealing the Moderating Role of Organizational Support in HR Professionals’ Competencies, Willingness, and Effectiveness Relationship: Empirical Evidence From a Developing Economy" was published in 2022. Journal: Front Psychol.

**Figure 3:** Structural model (direct hypotheses).

**Table 3:** Findings of the structural model.

	Original sample	Sample mean	Standard deviation	T statistics	Values of *p*
BA→HRPE	0.093	0.093	0.046	2.007	0.045
CA→HRPE	0.143	0.140	0.045	3.159	0.001
CCS→HRPE	0.10	0.098	0.07	1.434	0.152
HRPW→RPE	0.667	0.666	0.033	20.132	0.000
OE→HRPE	0.177	0.178	0.044	4.03	0.000
SA→HRPE	0.163	0.163	0.07	2.332	0.02
TMOD→HRPE	0.142	0.148	0.063	2.267	0.024
OS→HRPE	0.078	0.079	0.033	2.331	0.02
OS mod BA→HRPE	0.014	0.011	0.065	0.207	0.836
OS mod CA→HRPE	0.021	0.018	0.05	0.415	0.678
OS mod CCS→HRPE	−0.070	−0.078	0.060	1.152	0.250
OS mod HRPW→HRPE	0.027	0.038	0.072	0.375	0.708
OS mod OE→HRPE	0.202	0.208	0.051	3.969	0.000
OS mod SA→HRPE	0.161	0.157	0.075	2.136	0.033
OS mod TMOD→HRPE	0.121	0.124	0.062	1.941	0.05

Moreover, the moderation findings showed that organizational support positively and significantly moderates the relationships of HR Professionals’ Willingness (0.251^***^), Operational Executor (0.156^***^), Business Ally (0.214^***^), and Credible Activist (0.159^***^) with HR’s professional effectiveness (Figure 4). However, the organizational support showed weak but significant positive moderation between Strategy Architect and HR professionals’ effectiveness (0.099^**^). The moderating impact of organizational support remained negative and insignificant between Culture and Change Steward (−0.070), Talent Manager/Organization Designer (−0.023), and HR’s professional effectiveness.

**Figure 4:** Structural model (moderating hypotheses).

## Discussion

This study strived to unveil HR competencies and effectiveness under Ulrich’s Models of HR Competencies in Pakistan. This study has proved that HR professional’s competencies, including credible activists, talent manager/organization designer, strategy architect, operational executor, and business ally have a positive and significant impact on HR professional’s effectiveness in the Pakistani banking sector. Credible activist and operational executor were the most prominent contributing competencies to the HR professional’s effectiveness. These results have been in line with previous studies (Brachos et al., 2007; Grossman, 2007; Khatri et al., 2010; Morgan and Jardin, 2010).

The article "Revealing the Moderating Role of Organizational Support in HR Professionals’ Competencies, Willingness, and Effectiveness Relationship: Empirical Evidence From a Developing Economy" was published in 2022. Journal: Front Psychol.

Culture and change steward does not significantly and positively affect HR professionals’ effectiveness. This finding was consistent with Huselid et al (1997b), Ramlall (2006), and Ulrich et al (2008) about the significance of culture and change. These researchers argue that employee adjustment and culture significance bring success in the organizations only when organization fosters strong organizational culture and HR professionals nurture change in the organization (Tanure and Duarte, 2005). Business Ally and operational executors were also found to be positive and significant contributors toward HR professional’s effectiveness, which were proved by various illuminating studies (Long and Ismail, 2008; Ulrich et al., 2008; Payne, 2010). Furthermore, our results regarding the relationship between HR professionals’ willingness and HR professionals’ effectiveness were also positive and significant, which were consistent with the studies by Analoui (1999), Smith and McLaughlin (2004), Francis and Keegan (2006), and Ulrich and Grochowski (2012).

The study has introduced organizational support as a moderating variable among HR professionals’ competencies and HR professionals’ effectiveness. Findings show moderating relationship of organizational support is insignificant with most of HR professionals’ competencies. This finding was in line with Reilly (2012), who suggested that even in cases where HR professionals have the desire to contribute to organizational strategy, the lack of organizational support becomes an obstacle in doing so, which can intuitively affect the effectiveness of HR professionals.

## Managerial Implications

The present study’s findings are expected to enrich HR professionals’ understanding of HR professional competencies, which are essential contributors to their effectiveness, that ultimately impact their organizational performance. The performance of banks depends on attracting, managing, and motivating their employees, and the role of HR professionals’ competencies and their relationship with HR professional effectiveness is very significant. Moreover, HR, during normal conditions, does not take responsibility for the process of creating the strategy even it is known that strategy must be aligned with the latest HR practices. The present study will allow the HR professionals of the banking sector to be involved in strategizing for their organization.

Competition among banks and the demand for high-performing employees became a challenge for the HR department and its professionals. This research framework provides guidelines to HR professionals about what competencies are needed to enhance HR professional effectiveness. Eventually, the results of the study on HR professional effectiveness will hopefully relate to the improvement of the banking performance and the overall economic development of Pakistan.

The article "Revealing the Moderating Role of Organizational Support in HR Professionals’ Competencies, Willingness, and Effectiveness Relationship: Empirical Evidence From a Developing Economy" was published in 2022. Journal: Front Psychol.

As we know that banks provide service to their customers through employees. However, HR Professionalization is very crucial for effective services. In Pakistan, the banking sector is growing faster compared to other sectors; therefore, the level of competition is also increasing day by day. Every single bank tries to provide better services to their customers and get a competitive advantage over their competitors. Nevertheless, the study provides insights into the decision makers in the banking sector, which is that organizational support plays a vital role in enhancing the employee behavior toward their organization. Employee competencies are necessary skills to perform the task but employee willingness is something, which defines the overall script of the objectives or goals. Therefore, the top management should make strategies to channel the direction of the employees as well as increase their desire to work effectively and efficiently.

Furthermore, in the post-COVID-19 era, many challenges arise for the management to cope with them. One of the prior problems may be employees’ behavior toward their jobs. Due to the unclear situation prevailing in the global markets, employees’ willingness differs day by day because they are not sure about their job status. To overcome these fears, organizational support gives them the confidence to work with full of determination and willingness. As, the results of the study indicated that organizational support (moderating variable) significantly moderates the relationship between HR professional competencies, HR professional willingness, and HR professional effectiveness. Therefore, global organizations can get guidance from the results of the study and develop multiple strategies that increase organizational support.

## Theoretical Implications

The finding of this study has contributed to the existing body of knowledge by bringing new insights into the factors that may contribute to HR professionals’ effectiveness. This study has demonstrated the relationship between HR professional competencies, willingness, and moderating effect of organizational support on HR professional effectiveness in the context of the under-researched non-western organization using the resource-based view theory. Since most of the previous studies on HR professional competencies and their effectiveness had been tested in many countries like Malaysia, United States, Taiwan, and European Countries (Boselie and Paauwe, 2005; Han et al., 2006; Ulrich et al., 2007; Long and Ismail, 2008; Chaudhary et al., 2009). The results of those studies may not be applicable in the context of developing countries like Pakistan, Sri Lanka, and Bangladesh due to different research settings and unique national culture.

The article "Revealing the Moderating Role of Organizational Support in HR Professionals’ Competencies, Willingness, and Effectiveness Relationship: Empirical Evidence From a Developing Economy" was published in 2022. Journal: Front Psychol.

Moreover, this study as mentioned earlier tested a model Ulrich et al. (2009), which is based on HR performance theory and framework and has been well established in the human resource management field. The study, thus, adds to the existing body of knowledge by testing the applicability of the model in a new context and within a new set of environmental frameworks with additional benefits of theory development and refinement.

## Limitations and Future Directions

Despite various contributions, this study can also be viewed in the light of a few limitations which need to be recognized and may provide an indicator for future research efforts in this area. Firstly, this study’s context limits the generalizability of the results and may require future efforts to apply this research to other industrial sectors such as manufacturing and hospitality. Secondly, this study relied on self-reported questionnaire data; thus, the possibility of common method variance may exist since all the variables are measured using a single survey instrument. Thirdly, this study adopted a quantitative approach that might not explore human feeling or perceptions. Therefore, future studies should use a combination of both quantitative and qualitative approaches, such as in-depth interviews and focus group discussions, to provide validity of the findings of the study.

Fourth, the study considered the overall banking sector, in the future researcher can collect data from a single bank like Habib Bank Limited, United Bank Limited, Meezan Bank Limited, and many more working in the country for the reason that they have multiple branches operating in the country. It would give us deep insights into the local context because every city in a different province has a different culture. Fifth, the same theoretical model can be useful in the manufacturing sector as well, as in Pakistan the manufacturing sector contributes in very high numbers to the overall economy of the country.

## Data Availability Statement

The raw data supporting the conclusions of this article will be made available by the authors, without undue reservation.

## Ethics Statement

Ethical review and approval were not required for the study on human participants in accordance with the local legislation and institutional requirements. Written informed consent from the patients/participants or patients/participants legal guardian/next of kin was not required to participate in this study in accordance with the national legislation and the institutional requirements.

The article "Revealing the Moderating Role of Organizational Support in HR Professionals’ Competencies, Willingness, and Effectiveness Relationship: Empirical Evidence From a Developing Economy" was published in 2022. Journal: Front Psychol.

## Author Contributions

AA: data collection and analysis. MF: article drafting and literature review. MI: methods and conclusion. SS: discussion and proofreading. All authors contributed to the article and approved the submitted version.

## Conflict of Interest

The authors declare that the research was conducted in the absence of any commercial or financial relationships that could be construed as a potential conflict of interest.

## Publisher’s Note

All claims expressed in this article are solely those of the authors and do not necessarily represent those of their affiliated organizations, or those of the publisher, the editors and the reviewers. Any product that may be evaluated in this article, or claim that may be made by its manufacturer, is not guaranteed or endorsed by the publisher.
